The article "Evaluation Method of Public Physical Training Quality Based on Global Topology Optimization Deep Learning Model" was retracted in 2023. Reasons: signs of a paper mill; suspected computer-generated content; unreliable results or conclusions; concerns about the data.

# Evaluation Method of Public Physical Training Quality Based on Global Topology Optimization Deep Learning Model

**DOI:** 10.1155/2022/4043876

**Published:** 2022-09-15

**Authors:** JingMing Yan

**Affiliations:** School of Culture and Media, Xinhua University, Hefei 230088, China

## Abstract

In the quality evaluation of public sports training, the selected indicators are not comprehensive, resulting in some errors in the results of quality evaluation. Therefore, this paper designs a public sports training quality evaluation method based on the deep learning model of global topology optimization. Determine the basic principles of public sports training quality evaluation, determine the human coordinate points of public sports training by determining the basic section and basic axis of human training, and extract the data of public sports training quality evaluation. On this basis, quantify the public sports training quality evaluation index, construct the evaluation matrix, calculate the weight of the evaluation index, and determine the importance of the public sports training quality evaluation index. Preprocess the public sports training quality evaluation index set, search the optimal fitness value in the global topology optimization depth learning model, introduce the global topology optimization depth learning model, input the evaluation index and output the evaluation quality results, and realize the quality evaluation of public sports training. The experimental results show that the evaluation method in this paper can improve the accuracy of the evaluation results and is feasible.

## 1. Introduction

With the rapid development of the social economy, people's living standards are also improving, but people's physical fitness has been declining year by year. The emergence of this phenomenon makes people feel very surprising but also caused widespread concern from all walks of life. An important reason for the decline of people's physical quality is the lack of physical exercise [1]. Obesity, weakness, and other problems one after another become major obstacles to health. In the long run, the physical condition of the masses will eventually become an important issue affecting the development of the national physical condition. In order to promote the healthy development of the human body and improve the level of physical health, a large number of human and material resources are invested to organize and implement physical health tests [2]. However, in reality, these efforts have not achieved the expected effect, and instead, the resulting evaluation based on “physical health level” leads to social cognition deviation, false reported data of physical health tests, and many other problems [3]. Therefore, it is urgent to enrich and perfect the evaluation index system of mass sports fitness in China, whether from the needs of the times of sports fitness or from the needs of the country to promote the rapid development of sports fitness. The quality assessment of public sports training is to test the quality effect of public sports and is also an effective way to regulate the process of sports training [4]. It conducts a comprehensive and effective evaluation of the quality and process of public sports training, finds out problems in the process of public sports training, and promotes the further development of public sports training [5]. The significance of teacher training quality evaluation in traditional schools lies in the investigation of the basic situation and effectiveness of training work and the summary of experience through evaluation, so as to further improve training work and improve training effectiveness [6]. Therefore, it is of great significance to evaluate the quality of public physical training.

Therefore, relevant researchers have conducted a lot of research and achieved some results. Reference [7] proposed a method of physical education quality evaluation based on integration. Through the methods of literature research, interview, and field investigation, this paper explores the current evaluation of physical education quality, focuses on the analysis of theoretical research and practical needs, repositions from an integrated perspective, constructs a multiclassification system of physical education quality, and focuses on the real content of school physical education quality evaluation. The evaluation of physical education academic quality focuses on knowledge, ability, action, and health and systematically studies the respective evaluation points and the key points that should be grasped in the systematic setting of physical education quality evaluation standard. However, this method is more theoretical than practical. Reference [8] proposed an evaluation method of public sports service supply level from the perspective of basic public service equalization. The method used the entropy method to evaluate the single factor supply level and the comprehensive level of public sports service supply and used the exploratory spatial data analysis method to analyze the spatial distribution characteristics of the comprehensive level and single factor supply level of public sports service in China. The results show that this method can effectively evaluate public service facilities, but it cannot directly evaluate the quality of public sports training, and the results obtained are not practical. Reference [9] proposed an IPA-BASED public sports service quality evaluation model research. This method uses mathematical statistics and logical analysis method and IPA analysis method to design the evaluation model of public sports service quality and takes a certain national fitness center as the empirical object to test, in order to explore the path for the continuous improvement of public sports service quality in China. In this study, the public sports service quality evaluation scale covers five dimensions: availability, facility quality, health status, staff quality, and cost performance, with a total of 30 evaluation indicators. A total of 343 valid questionnaires were collected through the empirical test, which were reasonable in reliability and validity and suitable for quality evaluation. According to the coordinate region where the index evaluation results are located, the method can find problems and put forward improvement countermeasures for the national fitness center. IPA analysis method is suitable for the practical needs of public sports service quality evaluation in China and can be popularized and applied in a wider range. However, it needs to be improved by itself and further promoted with the integration of other quality management tools. Reference [10] proposed a public sports service quality evaluation method for large stadiums based on public perception. Based on the perspective of public perception and the modified SERVQUAL model, this method constructed the evaluation index system of public sports service quality in large stadiums and gymnasiums. Taking 2,685 valid questionnaires as sample data, the empirical research on the public sports service quality of 5 large stadiums in Hubei province is carried out by using AHP, fuzzy comprehensive evaluation, and TOPSIS method. However, this method has few indicators for sports training, so it is difficult to get accurate evaluation results.

Aiming at the problems in the above methods, this paper designs a new public sports training quality evaluation method based on the global topology optimization deep learning model. By determining the basic criteria for the quality evaluation of public sports training, the effectiveness of evaluation is improved; the quality data of public sports training is extracted; the quality evaluation indicators of public sports training are constructed; the indicators are normalized; and the quality evaluation of public sports training is realized by using the global topology optimization deep learning model. The results show that the proposed method can effectively improve the accuracy of the evaluation results and has certain feasibility.

## 2. Evaluation Principles and Index System Construction of Public Sports Training Quality

### 2.1. Principles of Public Sports Training Quality Evaluation

#### 2.1.1. Principle of Subjectivity

The principle of subjectivity means that the responsible subject must be clear in the quality evaluation of public sports training. Students are the main body of public sports training quality evaluation. In the process of evaluation, we should enhance the consciousness of the quality subject. The construction of the evaluation system should fully consider the main role of students, establish and improve the quality evaluation system, and improve the evaluation quality. Give play to the main role and continue to improve the quality of public sports training.

#### 2.1.2. Objective Principle

The goal principle means that the quality system of public sports training should be consistent with the training purpose. The ultimate goal is to improve the quality of public sports training [11]. The objective principle requires the evaluation to pay attention to the establishment, guarantee, and implementation of project objectives.

#### 2.1.3. Systematic Principle

The systematic principle refers to that all parts of the quality evaluation of public sports training are interrelated and interactive. To give full play to the overall advantages of evaluation, we must proceed from the whole and deal with it comprehensively. The part is the constituent element of the whole. The part should obey the whole. Any decision should not violate the overall goal of strategic decision-making.

#### 2.1.4. Scientific Principle

The scientific principle refers to the construction of public sports training quality evaluation system to select the most characteristic and representative influence factors, select the most widely used index and the best response system on the basis of scientific research, optimize it to the simplest and best, and form the most scientific index system [12].

#### 2.1.5. Principle of Feasibility

The principle of feasibility means that the scheme chosen in the construction of public sports training quality evaluation system cannot exceed the subjective and objective conditions. First of all, the evaluation index can use the corresponding sentences to explain its contents, get the corresponding data through the corresponding measurement tools and draw a clear conclusion, and use the principle of quantitative index measurement as the main and qualitative index measurement as the auxiliary. Therefore, based on the scientific demonstration of various possible schemes, we should pursue the simplicity of scheme implementation.

### 2.2. Data Extraction of Public Sports Training Quality Evaluation

In order to realize the effective evaluation of public sports training quality, it is necessary to clarify the relevant data of public sports training quality evaluation, that is, it is necessary to extract the data on human public sports training quality [13]. In order to facilitate the description and analysis of public sports, the basic plane and basic axis of the human body are usually defined in the standard upright position, as shown in Figure 1.

The basic plane of the human body includes sagittal, coronal, and horizontal planes, which are perpendicular to each other. Among them, the sagittal plane is a vertical section in the fore-and-aft direction, which divides the body into left and right parts along the fore-and-aft direction of the human body; coronal plane, also known as the frontal plane, is a vertical section in the left and right directions and divides the body into front and back parts along the left and right directions of the human body; and horizontal plane, also known as cross-section, is parallel to the ground and divides the body into upper and lower parts. The basic axes of the human body include sagittal, coronal, and vertical axes, which are perpendicular to each other [14]. Taking different basic axes of the human body as the tangent point, the relevant data on public sports training quality are determined. In human training data extraction, the relevant motion information data is extracted with the help of a camera. First, the five-parameter model of a linear camera is determined as follows:

(1) $$\begin{array}{c} \left[\begin{array}{c} \bar{a}\\ \bar{b}\\ 1 \end{array}\right]=p_{i}\left[\begin{array}{c} \frac{a_{c}}{z_{c}}\\ \frac{b_{c}}{z_{c}}\\ 1 \end{array}\right]=\left[\begin{array}{ccc} f_{x} & f_{s} & u_{0}\\ 0 & f_{y} & v_{0}\\ 1 & 1 & 0 \end{array}\right]. \end{array}$$

The matrix *p*_*i*_ is the internal parameter matrix under the linear model of the camera, making two sets of translation movements in three-dimensional space and controlling the attitude of the camera for self-calibration; (*f*_*x*_, *f*_*y*_) is the magnification coefficient of the image plane in the *X*-axis direction and the *Y*-axis direction: (*u*_0_, *v*_0_). Main point coordinate: *f*_*s*_ is the coupling amplification coefficient when the *X*-axis and the *Y*-axis are not perpendicular;

The nonlinear model formula of the camera for extracting human training data is then determined as follows:

(2) $$\begin{array}{c} \left\{\begin{array}{c} \bar{a}=a+D_{a}\left(a,b\right),\\ \bar{b}=b+D_{b}\left(a,b\right), \end{array}\right. \end{array}$$

where $\left(\bar{a},\bar{b}\right)$ is the human training image point coordinate under the linear model, (*a*, *b*) is the actual human training image point coordinate, and (*D*_*a*_, *D*_*b*_) represents the nonlinear distortion value.

The nonlinear model camera imaging of the same target training point at multiple different human training viewpoints is set to *S*^(0)^, *S*^(1)^,…, *S*^(*n*)^, and the feature matching point in the extracted human training is set to

(3) $$\begin{array}{c} \left(S_{j}^{\left(i\right)},S_{i}^{\left(i\right)},1\right)\in S^{\left(i\right)},\;i=1,2,3\ldots n. \end{array}$$

According to the determined characteristic matching points in human training, the training movement coordinates of different points in human training are determined as follows:

(4) $$\begin{array}{c} \left\{\begin{array}{c} {\bar{x_{j}}}^{\left(i\right)}=x_{j}^{\left(i\right)}+S_{x}\left(x_{j}^{\left(i\right)},y_{j}^{\left(i\right)}\right)\\ {\bar{y_{j}}}^{\left(i\right)}=y_{j}^{\left(i\right)}+S_{y}\left(x_{j}^{\left(i\right)},y_{j}^{\left(i\right)}\right) \end{array}\right.,\;i=1,2,3,\ldots \end{array}$$

Finally, matching human training points in public sports training and extracting public sports training quality assessment data requires a series of processing of images acquired by two cameras set side by side, and obtaining depth information, which has very important applications in robot navigation, three-dimensional reconstruction, and other fields. The stereo matching assumes that two cameras are identical and the optical axes are parallel with only lateral displacement between cameras. In the paired images, the pole line is parallel to the *x*-axis, and and horizontal state is maintained [15]. Since a completely ideal stereo camera configuration is difficult to achieve, feature detection, description, and sparse feature matching are required, that is, stereo correction to meet the assumed conditions of stereo matching. Here, feature detection is used to identify more obvious visual features that recur in multiple views. Such sparse features require a corresponding feature description for matching so that feature detection allows images from cameras with different viewpoints and different parameters. Get

(5) $$\begin{array}{c} E\left(p,q\right)=\exp\left(-\frac{\Delta_{c}\left(I_{0}\right.\left(p\right),I_{0}\left(q\right)}{\gamma_{c}}-\frac{\Delta_{g}\left(p,q\right)}{\gamma_{g}}\right), \end{array}$$

where *E*(*p*, *q*) is human training points in public sports training, *γ* represents the weight value of stereo matching, and *g* represents the similarity value of sports training data.

In the process of extracting public sports training quality evaluation data, the basic section and basic axis of human training are determined, the human coordinate points of public sports training are determined through the five parameter model, and the evaluation of public sports training quality evaluation data is completed through three-dimensional matching and coefficient characteristics. Based on the relevant data of evaluation, it is convenient to carry out subsequent research.

### 2.3. Construction of Public Sports Training Quality Evaluation System, That Is, Quantitative Research on Indicators

Based on the data extraction of public sports training quality evaluation, this paper takes these data as the research object to construct indicators and quantify them. First, build a public sports training quality evaluation system. The establishment of public sports training quality evaluation index system needs to be based on the guiding ideology and working principles of the evaluation work. In addition to considering the main characteristics of the training project, it should also be combined with the project characteristics and various qualities and abilities that teachers should have [16]. This paper classifies and analyzes the factors affecting the public sports training quality evaluation system and the professional characteristics of teachers and, combined with expert interview opinions, divides the factors affecting the public sports training quality into four major aspects, namely the first-class indicators of the evaluation system: training resources, training scheme, training process, and training effect. See Figure 2 for details.

For the evaluation of public sports training quality, there are many influencing factors. Therefore, in the evaluation of public sports training quality, it has a certain fuzzy attribute, which is a more important part of the evaluation results. Therefore, this paper will introduce the combination of the fuzzy comprehensive evaluation method and the deep data mining method to determine the membership of the evaluation index of public sports training quality [17].

To quantify the evaluation indexes of public sports training quality through the fuzzy comprehensive evaluation method, it is necessary to construct the influencing factor set, evaluation set, and membership degree of relevant influencing factors of public sports training quality evaluation indexes. The influencing factor set of evaluation indexes is as follows.

Then, we construct the membership subset of the public sports training quality evaluation indicators, namely

(6) $$\begin{array}{c} L_{i}=\left\{l_{i1},l_{i2},l_{i3},\ldots l_{\text{in}}\right\},\\ V_{i}=\left\{v_{i1},v_{i2},v_{i3},\ldots v_{\text{im}}\right\}, \end{array}$$

where *L*_*i*_, *V*_*i*_ represents the specific membership set corresponding to the first index (or the teaching performance of a certain subject) corresponding to the related evaluation index of public sports training quality. At this time, the membership calculation formula of the specific public sports training quality evaluation index is as follows:

(7) $$\begin{array}{c} F_{\left(L_{i},V_{i}\right)}=\frac{P_{i}}{q_{i}}, \end{array}$$

where the value range of the lower angle mark is 1,2,…. *P*_*i*_ is used for the specific index level and *q*_*i*_ is used to represent the total number of participants participating in the public sports training quality evaluation.

After the scalarization of the above public sports training quality evaluation index, the weight calculation of the evaluation index is needed. The evaluation matrix is represented as *W*. The above evaluation indexes all have a subset of evaluation membership; all influencing factors are set as one; and the evaluation matrix of the evaluation index is constructed in the feasible domain of influence factors [18]. The membership value of the evaluation index of public sports training quality is obtained by normalization processing [19]. The calculation process is as follows:

(8) $$\begin{array}{c} W=\left\{\begin{array}{cccc} w_{11} & w_{12} & \ldots & w_{1n}\\ w_{22} & w_{22} & \ldots & w_{2n}\\ \ldots & \; & \; & \;\\ w_{n1} & w_{n2} & \ldots & w_{nn} \end{array}\right\}. \end{array}$$

In order to improve the accuracy of the public sports training quality evaluation index, the membership degree and the evaluation membership degree value are calculated repeatedly to obtain the evaluation value of the impact index. The quantitative evaluation index of public sports training quality is obtained, and the fuzzy comprehensive evaluation results are as follows:

(9) $$\begin{array}{c} S\times W=\left(S_{1},S_{2},\ldots S_{N}\right)\left[\begin{array}{c} w_{1}\\ w_{2}\\ \ldots \\ w_{3} \end{array}\right]. \end{array}$$

At the same time, the effectiveness of the evaluation is improved according to this result. The quantitative process of public sports training quality evaluation indicators is shown in Figure 3:

In the quantification of public sports training quality evaluation indicators, the public sports training quality evaluation indicators are quantified by the combination of a fuzzy comprehensive evaluation method and deep data mining method. On this basis, the evaluation matrix is constructed to calculate the weight of evaluation indicators and determine the importance of public sports training quality evaluation indicators, so as to lay a foundation for follow-up research.

## 3. Implementation of Public Sports Training Quality Evaluation Based on Global Topology Optimization and Deep Learning Model

Public physical training quality evaluation is the measurement, analysis, and evaluation of the quality of physical education teaching. It takes the process and results of the organic combination of teaching objectives, teaching contents, teaching methods, and other factors involved in teaching activities as the evaluation object. It is the evaluation of the overall function of teaching activities. It is assumed that the evaluation of public physical education training and teaching mainly includes the evaluation of students' physical education academic achievement and the evaluation of physical education curriculum teaching quality. In the comprehensive evaluation of the teaching quality of public physical education in colleges and universities, we should determine the elements of evaluation and the specific evaluation contents scientifically and reasonably. In other words, a physical education teaching quality evaluation system should be determined. The evaluation index is the basic unit of the evaluation system and a relatively fixed parameter.

Based on the evaluation index system and quantification of public sports training quality, this paper designs an evaluation algorithm based on global topology optimization deep learning model to achieve the goal of this paper. Deep learning is a new research direction in the field of machine learning. It is introduced into machine learning to make it closer to the original goal: artificial intelligence. Deep learning is the internal law and representation level of learning sample data. The information obtained in the learning process is very helpful to the interpretation of data such as text, images, and sound. Its ultimate goal is to make the machine have the ability to analyze and learn like human beings and can recognize characters, images, sounds, and other data. Topology optimization is a branch of structure optimization. Structural optimization design was developed in the 1960s. It combines engineering design problems with mathematical optimization methods and produces a method that can solve the optimal engineering problems. According to the different variables of structural topology optimization design, the structural optimization design can be divided into three parts: size optimization, shape optimization, and topology optimization [20]. Among the three, topology optimization is the most challenging and practical direction in the current optimization design methods. This structure combines with a deep learning algorithm to form a more advanced training algorithm. Therefore, this paper adopts the global topology optimization depth learning model to realize the quality evaluation of public sports training [21]. The basic structure of the global topology optimization deep learning model is shown in Figure 4:

The global topology optimization depth learning model is composed of two dense connection layers and four transposed convolution layers. Its output result is the quantitative index data of public sports training quality evaluation obtained above, and the obtained result is the research result [22].

According to the global topology optimization depth learning model set above, determine the state of quantitative indicators for public sports training quality evaluation and effectively evaluate the quality of public sports training [23]. The specific process of public sports training quality evaluation is as follows:

**Step 1 .**

Through the global topology optimization, the smoothing factor in the neural network in the deep learning model is the optimization goal, and the optimal model of index evaluation is constructed [24]. Set and initialize the evaluation index data of public sports training quality as follows:

(10) $$\begin{array}{c} T=\left\{t_{i},i=1,2\ldots n\right\}. \end{array}$$

The public sports training quality evaluation index is divided into a training set and a test set defined as follows:

(11) $$\begin{array}{c} T_{\text{train}}=\left\{t_{1},t_{2},\ldots t_{n}\right\},\\ T_{\text{test}}=\left\{t_{m+1},t_{m+2},t_{m}\right\}m<n. \end{array}$$

Then, according to the division of the training set, the zero mean standardization method is used to preprocess the public sports training quality evaluation index set, and the following results are obtained [25]:

(12) $$\begin{array}{c} T_{\text{train}}^{\prime }=\frac{t_{t}-\sum_{t=1}^{m}t_{t}/m}{\sqrt{{\sum_{t=1}^{m}\left(t_{t}-\sum_{t=1}^{m}t_{t}/m\right)}^{2}/m}}. \end{array}$$

**Step 2 .**

Initialize the parameters of the preprocessed training set and randomly generate the initial neurons according to the size [26], location, and population size of neurons in the global topology optimization deep learning model. The neuron set is obtained as follows:

(13) $$\begin{array}{c} C=\left|c_{1},c_{2},\ldots c_{n}\right|. \end{array}$$

**Step 3 .**

Calculate the fitness value by integrating constraints and fitness function according to the randomly generated initial neuron set as follows:

(14) $$\begin{array}{c} Z=\frac{T_{\text{train}}^{\prime }}{1+C}. \end{array}$$

**Step 4 .**

According to the calculated fitness value, search for the optimal fitness value in the global topology optimization deep learning model, that is, *y*_*i*_, the minimum error value erro_*i*_ between the actual quality value *β*_*i*_ and the public sports training quality evaluation index at *i* time from the prediction starting point, whose expression is as follows:

(15) $$\begin{array}{c} {\text{erro}}_{i}=\frac{1}{n}\sum_{i=1}^{n}\frac{\left|\beta_{i}-y_{i}\right|}{y_{i}}\times 100\%. \end{array}$$

**Step 5 .**

Check the conditions for exiting the program to reach the maximum number of iterations or meet the convergence accuracy. If so, output the best result.

**Step 6 .**

Update the speed and position of neurons according to the current overall fitness value and individual fitness value.

**Step 7 .**

Use the modified linear unit to obtain the construction operation function, that is,

(16) $$\begin{array}{c} \eta_{i+1}=\max\left(0,v_{i}\times k_{i+1}+v_{j}\right), \end{array}$$

where *k*_*i*+1_ describes the evaluation index value obtained when the model network layer, *t*_*i*_ describes the weight value obtained when the convolutional layer is used, and *v*_*j*_ describes the deep learning network bias parameter, represents the maximum extreme of the running function, and selects the maximum extreme method.

(17) $$\begin{array}{c} k_{i+1}=\max y_{i}. \end{array}$$

**Step 8 .**

Extract the optimal value obtained from the model and use the optimal parameters to establish a global topology optimization depth learning model as follows:

(18) $$\begin{array}{c} R\left[g^{2}\right]=\varphi R{\left[g^{2}\right]}_{t+1}+z\left(1-\varphi \right)\beta_{i}, \end{array}$$

where *z* represents the gradient at time *t* and *φ* represents the coefficient of the expected value of *g*^2^.

**Step 9 .**

Enter the training sample data into the global topology optimization deep learning model to train the model. Input the test data into the trained model, output the evaluation quality results in the output layer *P*, and complete the quality evaluation of public sports training as follows:

(19) $$\begin{array}{c} U_{P}=R{\left[g^{2}\right]}_{t}h, \end{array}$$

where *U*_*p*_ represents the state of the neural network memory module and *h* represents the output of the memory module.

In the implementation of public sports training quality evaluation, the zero mean standardization method is used to preprocess the public sports training quality evaluation index set, search for the optimal fitness value in the global topology optimization deep learning model, introduce the global topology optimization deep learning model, input the evaluation index, and output the evaluation quality results.

## 4. Experimental Analysis

### 4.1. Experimental Environment and Parameter Setting

The algorithm design in this experiment is based on the framework of PyTorch 1.2.0, Ubuntu 18.04 system, and two Titan-RTX 16g graphics cards. The network of global topology optimization deep learning model was trained for 50 times of generation selection, and the learning rate of different iterations was changed 0.2 for iteration 1, 0.01 for iteration 60, 0.001 for iteration 80, and 0.0001 for generation 100, and the batch size was set to 1. In the process of public sports training, the samples of full marks of test actions in training data sets are input into the conditional network for training, and various test action template information (feature layer parameters at the last layer of the network) is obtained. Then, this information is used as conditional input, and the score category prediction network is separately trained. The second method is to input all test action samples in the training set into the conditional network for training without screening and then train the score category prediction network separately. In the experiment, students of a physical education major class in a university were selected as the research object. There were 50 middle school students in the class, and 30 students were randomly selected as the experimental object. Experimental analysis was conducted on the public physical education training programs, teaching contents, and training effects of this major in our school. Thirty people were divided into two groups: one for the experimental group and the other for the control group. The environment and conditions in the experiment were consistent, and the error value of the evaluation was reduced. The schematic diagram of the training objectives of specific experimental subjects was shown in Figure 5.

### 4.2. Analysis of Experimental Results

Based on the set experimental environment and relevant parameters, an effective evaluation of the quality of public sports training is carried out. In the experiment, the satisfaction of 30 people in training is investigated to determine whether the selection of experimental indicators determined by this method meets the wishes of the tester. According to the evaluation index of teaching quality of public physical training courses in Table 1, the quality of public physical training is studied.

Based on the contents of Table 1, the statistical results of training quality satisfaction of sample objects are shown in Table 2.

It can be seen from Table 2 that in addition to the objective and realistic conditions, the subjective feelings of the students are also an important basis for evaluation. Students are also the audience, and their satisfaction with public sports training is a direct reflection of the training quality. As can be seen from the data in Table 2, the training facilities have the highest satisfaction level, with the basic satisfaction level above 70%, from which it can be seen that the evaluation indicators selected in this paper have certain feasibility.

In order to further highlight the effectiveness of this method, the experiment compares the accuracy of the sample public sports training quality data evaluation by comparing this method, reference [7] method, and reference [8] method many times and measures the accuracy results of the three methods on the sample public sports training quality data evaluation. The results are shown in Figure 6.

By analyzing the experimental results in Figure 6, it can be seen that there are some differences in the accuracy of sample public sports training quality data evaluation by using the methods of this paper, reference [7], and reference [8]. Among them, the accuracy of this method in the evaluation of sample public sports training quality data is higher than the other two methods, and the performance is always relatively stable, higher than 90%, while the evaluation accuracy of the other two methods is lower than that of this method. Therefore, it can be seen that the evaluation effect of this method is better.

On the basis of ensuring the accuracy of the above sample public sports training quality data evaluation, the experiment further verified the time cost of this method, reference [7] method, and reference [8] method for the sample public sports training quality data evaluation. The results are shown in Figure 7.

By analyzing the experimental results in Figure 7, it can be seen that there are some differences in the time cost of evaluating the sample public sports training quality data by using the methods of this paper, reference [7], and reference [8]. Among them, from the trend of the curve, the evaluation time of this method is shorter, while the evaluation time of the other two methods is longer. In contrast, the evaluation speed of this method is faster, which verifies the effectiveness of this method.

## 5. Conclusion

This paper designs a public sports training quality evaluation method based on the global topology optimization depth learning model. Determine the basic principles of public sports training quality evaluation, determine the basic section and basic axis of human training, use the linear camera to determine the human coordinate points of public sports training through the five parameter model, and complete the data extraction of public sports training quality evaluation through three-dimensional matching and coefficient characteristics. On this basis, through the combination of fuzzy comprehensive evaluation method and deep data mining method, the evaluation indexes of public sports training quality are quantified. On this basis, the evaluation matrix is constructed to calculate the weight of the evaluation indexes and determine the importance of the evaluation indexes of public sports training quality. The zero mean standardization method is used to preprocess the public sports training quality evaluation index set, search the optimal fitness value in the global topology optimization deep learning model, introduce the global topology optimization deep learning model, input the evaluation index and output the evaluation quality results, and realize the quality evaluation of public sports training. Although this paper has improved the evaluation accuracy in this study, the evaluation indicators are still incomplete. In the next step, I will continue to explore the evaluation indicators to improve the shortcomings of this method.

## Figures and Tables

**Figure 1:** Schematic diagram of basic section and basic axis of the human body.

**Figure 2:** Schematic diagram of public sports training quality evaluation index system.

**Figure 3:** Quantitative process of public sports training quality evaluation index.

**Figure 4:** Basic structure of global topology optimization deep learning model.

**Figure 5:** Schematic diagram of public sports training objectives of experimental subjects.

**Figure 6:** Accuracy analysis of public sports training quality data evaluation with different methods.

**Figure 7:** Comparison of time cost assessed by different methods.

**Table 1:** Evaluation indicators of teaching quality of public physical training courses.

Index	Content	Evaluation grade	Weight
Content of courses	Whether it is in line with students' reality and pays attention to students' personality development	Excellent	0.098
Teaching attitude	Prepare before class, communicate with teachers and students in class, and answer patiently after class	Excellent	0.092
Teaching method	Explain clearly, stimulate students' interest in sports, and mobilize students' learning enthusiasm	Excellent	0.096
Teaching effectiveness	Whether the lectures are vivid and attractive so that students' subjectivity can be brought into play	Excellent	0.095

**Table 2:** Statistical results of training quality satisfaction of sample objects (%).

Index	Very satisfied	Satisfied	Commonly	Unsatisfied	Very dissatisfied
Training facilities	62.12	30.14	4.56	3.18	0
Training resources	42.25	32.54	9.63	15.58	0
Training conditions	43.21	33.69	4.21	18.89	0
Dietary conditions	52.14	32.14	5.23	10.49	0
Training content	59.63	26.52	5.21	8.62	0
Training effect	54.32	32.14	4.96	8.58	0

## Data Availability

The raw data supporting the conclusions of this article will be made available by the author, without undue reservation.
